# The Public Sentiment Analysis of Double Reduction Policy on Weibo Platform

**DOI:** 10.1155/2022/3212681

**Published:** 2022-09-08

**Authors:** Weichen Jia, Jun Peng

**Affiliations:** ^1^School of Media and Law, Ningbo Tech University, Ningbo 315000, China; ^2^School of Education, City University of Macau, Macau 999078, China

## Abstract

Weibo platform is an indispensable transmission channel in education policy release and dissemination. The events and sentiments contained in education policies microblogs include the public sentiment and support the general management and guidance scientifically and efficiently. This study constructs a dataset based on the “Double Reduction Policy” relevant microblogs and comments. The policy events are extracted by Latent Dirichlet Allocation (LDA) model and Language Technology Platform (LTP). Based on the emotion dictionary, an attention-based BiLSTM model is constructed to classify the public sentiments. The experimental results reveal four themes: “industry impact,” “institutional supervision,” “public feedback,” and “policy implementation.” The distribution conforms to the development trend of online public sentiments.

## 1. Introduction

Chinese authorities have introduced a set of guidelines to ease the burden of excessive homework and off-campus tutoring for students undergoing compulsory education (Double Reduction Policy) on May 21, 2021 (General Office of the Communist Party of China Central Committee and the State Council General Office, 2021). This document requires strict governance and norms than the outside training behavior comprehensively. Social network platform like the Weibo platform has become an indispensable transmission channel in policy dissemination and audient reflection. With the policy promotion continuing, the number of news and comments on the Weibo platform are increasing, and the public sentiments is generating various reaction. This study displays the event and emotion portraits based on the “Double Reduction Policy's” relevant microblog and comments below. Then analysis of the emergence of social reflect and influence on public sentiment since the policy was promulgated. The interpretation could provide strong support for the education department to grasp the situation of public sentiments and promote the “Double Reduction Policy” scientifically and efficiently.

## 2. Related Work

This study regards the network public sentiment lifecycle, “Double Reduction Policy” events portrait, and public sentiment as the object of study. This section will review the research progress of these objects.

### 2.1. Network Public Sentiment and Lifecycle

Researchers construct their definition of network public sentiment from different aspects, such as the event object (government policy, social hot spot), and public reaction (event cognition, opinion, behavior) [1–8]. This study regards the network public sentiment as the sum of public awareness, attitude, and activities by different groups. The subject of network public sentiment is the masses, and the object is the social events, which mean the primary expression of public sentiment is focused on popular psychology, and the public sentiment could extend to various social events. So that the network public sentiment could reflect the people's social and political attitudes toward organizing the class. In the convergence media era, network public sentiment possesses the characteristic of viral transmissions, such as fast speed, widespread, and significant influence. These features put forward higher requirements for the researchers and managers to have a clearer control of network public sentiment. The lifecycle of network public sentiment is an essential part of research in this era as mentioned above. This lifecycle study could support the construction of measures and governance models. Researchers could provide corresponding methods and strategies based on the laws and characteristics of different stages of network public sentiment.

Scholars raise various methods to divide the network public sentiment lifecycle [9, 10]. The main difference is the late-stage (decline and termination stage). Some scholars subdivide the decline stage of the life cycle of network public sentiment into the repeated stage, fade stage, and long tail stage [5], and some simply define it as the decline stage [1]. This study defines the network public sentiment lifecycle into four stages, which contain generation stage, outbreak stage, extinction stage, and long tail stage. The division algorithm of lifecycle is different. Traditional lifecycle division usually adopts manually operated ones based on visualization time-series data [1, 11]. The advantage of traditional lifecycle division is simple and intuitive, but it also has problems of roughness and low efficiency. The quantitative division could acquire the characteristics of each lifecycle stage through information entropy, machine learning algorithm, and deep neural network, and achieve a good performance [6, 7, 12–14].

### 2.2. Event Extraction

The event extraction is regarded as an important technology in the field of network public sentiment monitoring. It is a data process technology, which could extract event types and elements from unstructured text, including event information by natural language processing technology, and present the event in a structured form. The transformation of network public sentiment is always triggered by social events. The event extraction technology could figure and reveal the hot/emergency event in the first time and provide support for predicting changes.

The event extraction technology includes two trends: pattern match and machine learning.

The pattern match method is developed from the rule-based match method. The core of these match strategies is the construction of matching rules. Researchers develop a great deal of domain-based knowledge databases manually to support the knowledge maps. Representative studies include the CIRCUS for conceptual sentence analysis proposed by Lehnert in 1990 [15], AutoSlog proposed by Ellen, and PALKA presented by Kim and Moldovan [16], and TwiCal presented by Ritter et al. [17]. The technology of knowledge dictionary has been updated (from manual to automated). However, they are still established based on language patterns, such as concept nodes, sematic framework, phrase structure, and lexical information [18, 19]. Event extraction based on the pattern match method could achieve a sound performance in specific corpora, but this method has a weak generalization ability. The rules need to be updated in a new domain to ensure the performance of the model does not affect by text noise.

To avoid the shortcomings of pattern match method, researchers try to adopt machine learning for event extraction. This method consists of shallow and deep neural networks. The core of these match strategies is the classification model. These models could recognize the events in the corpus.

The event extraction constructed by a shallow neural network focus on the Named Entity Recognition (NER) and event classifier. They could recognize and classify the event information, trigger words, elements, from the corpus [20]. The maximum entropy (ME) model and conditional random field (CRF) model become mainstream technologies. Researchers are used to splitting the extraction task into the event trigger words recognition and event elements recognition [20], and adopt different algorithms for the corresponding subtask. ME model is mainly used to construct the NER framework, event element recognition, and classifier construction [21, 22]. CRF technology is used to segment words and semantic role annotation [23–26]. The shallow neural network could reduce the dependence on domain experts, but it needs the support of large-scale annotated training corpus. The cost of corpus construction makes researchers turn to the deep neural networks. The event extraction method based on a deep neural network converts the annotated training data into vectors and input into the neural network for calculation. The neural network could extract the semantic features automatically.

To achieve these tasks, researchers mainly focus on dataset annotation, language model, and model structure. Researchers adopt convolutional neural network (CNN)/recurrent neural network (RNN) with machine learning model to construct a mixed model to optimize the basic functions of event extraction such as part of speech tagging and named entity recognition [27–29]. Some researchers also use word vector (Word2vec, Bert) to achieve better performance [26, 30]. Deep neural networks could migrate to different fields quickly without building domain knowledge maps and annotating corpora.

### 2.3. Text Sentiment Analysis

Text sentiment analysis is a necessary component in network public sentiment analysis. It could understand, explain, and predict network public sentiment [31]. The dictionary-based analysis and deep learning classifier become the mainstream technologies.

Dictionary-based sentiment analysis adopts algorithms to identify emotional vocabulary and corresponding sentence structures, and calculate sentiment scores based on the emotional corpus. For the differences in language pattern, this method is very dependent on domain corpus [8], sentiment analysis needs to be adjusted according to the field of domain. Researchers mainly focus on the construction of sentiment dictionary and the optimization of calculation methods. Some researchers combine sentiment dictionary with the LDA model and PMI algorithm [32, 33]. The advantage of dictionary-based analysis is that it does not require training data and the calculation speed is fast. However, this method cannot obtain context information, and it is complex to update the dictionary when new words appear in the corpus.

The method based on deep learning is transforming the calculation task of sentiment score into a classification task to identify different sentiments. This process method mainly contains machine learning algorithm classification and deep neural network classification.

The machine learning trend includes unsupervised learning, semisupervised learning and supervised learning. SVM, LDA, ME, and other shallow neural network models and their variants are used to classify the input corpus. The differences are in whether training data are annotated [34]. Semisupervised learning is widely used in sentiment analysis of Twitter and Weibo, because such short texts generated based on social network have a large amount of unannotated dataset [35–37]. The disadvantage of this trend is the requirement of annotation, which is time-consuming and labor-intensive, and has some problems such as inconsistent labeling.

The deep neural network trend has been widely used in sentiment analysis [34]. CNN and RNN (including varieties BiLSTM and GRU) are the most widely used structures. Researchers usually adopt word-embedding technology combined with RNN structure (LSTM and BiLSTM) to achieve better performance [34]. However, the size of RNN is larger than CNN, which might lead to a longer training time. At the same time, deep neural networks have a huge demand for training datasets [38]. In sentence-level sentiment analysis of Twitter and Weibo, researchers import attention mechanism to achieve more accurate sentiment classification by constructing attention-based LSTM or BiLSTM network [38–41].

## 3. Data Source and Method

### 3.1. Data Collection and Preprocess

The aforementioned shows that the network public sentiment has its lifecycle. To achieve the whole “Double Reduction Policy” event, this study set the time span from the generation stage to the long tail stage.

According to the “Microindex”^1^, the number of relevant microblog was below 50 for 9 consecutive days after October, which indicates the lifecycle has been in the extinction stage.

The time span is “July 1, 2021 to October 16, 2021,” we adopt a python^2^ script to construct the microblog public sentiment dataset of the “Double Reduction Policy” event (hereinafter referred to as the dataset). This dataset includes 10155 microblog relevant to “Double Reduction Policy” or “Double Reduction” topic, and 22463 comments. We clean the text in the dataset, the data cleaning rule is shown in Table 1.

After the preprocessing, this study adopts the LTP^3^ [42] to preprocess (clause, word segmentation, tagging) the cleaned dataset.

### 3.2. Method

#### 3.2.1. Framework

Research framework includes descriptive analysis of “Double Reduction Policy” events, events clustering analysis, public sentiment analysis, and interpretation of the influence.

In the descriptive analysis, we divide the “Double Reduction Policy” lifecycle based on the qualitative method, and visualize a regional heat map based on public attention. In the clustering analysis, we cluster the event and filter the event trigger vocabulary through the LDA model and LTP. Then classify the microblog and comments based on the analysis result. In the public sentiment analysis, this study classifies the public sentiment according to DUTIR^4^ classification, and construct an attention mechanism based two-way long- and short-term memory network (Attn-BiLSTM) model to calculate the sentiment score. We could reveal the distribution of public sentiment based on the calculate result.

#### 3.2.2. Clustering Analysis of “Double Reduction Policy” Events

1. The microindex is an index based on the amount of mention, reading, and interaction; this index could reflect the popularity of keywords on Weibo platform.
2. Python is a programming language that lets you work more quickly and integrate your systems more effectively.
3. Language Technology Plantform, LTP is an open-source neural Chinese Language Technology Platform with pretrained models.
4. DUTIR is a Chinese ontology resource sorted and marked by the information Retrieval Office of Dalian University of Technology. This resource describes a Chinese word (phrase) from word class, emotional category, emotional intensity, polarity, and the forth.

This study adopts LDA model to generate event cluster. The dataset is classified into “industry impact,” “institutional supervision,” “public feedback,” and “policy implement.” We generate the keywords list of each topic, and label the part of speech (Pos) by LTP. The events clustering is based on the trigger words, filtered through the annotation and classification.

#### 3.2.3. Public Sentiment Analysis

In the DUTIR design, the sentiment-relevant vocabulary is divided into seven categories, including optimism, beauty, anger, sadness, fear, disgust, and shock. This study analyzes the public sentiment in “Double Reduction Policy” events based on dictionary method and deep learning network. We calculate the emotional intensity of corpora related to “Double Reduction Policy” through the DUTIR and a modifiers dictionary. The emotional intensity should calculate the negative words and of adverbs, respectively. The emotional intensity formula is shown in formula (1):

(1) $$\begin{array}{c} E_{i}={\left(-1\right)}^{o_{i}}*\alpha_{i}*\beta_{i}*m. \end{array}$$

The *E*_*i*_ represents the final sentiment score, o_i_ represents the frequency of negative words, *α*_I_ represents the score of the index *i* adverb, *β*_I_ represents the score of index *i* emotional word, m represents the weight of the corresponding couple.

First, text in the dataset is transformed into vector, a word2vector model of “Double Reduction Policy” dataset is constructed. Second, we adopt algorithm based on dictionary and an Attn-BiLSTM model to process the word2vector model, respectively. Finally, we achieve the public sentiment distribution of “Double Reduction Policy” events.

A bidirectional long and short-term memory network (Attn-BiLSTM model) based on attention mechanism is adopted in this study, as shown in Figure 1. The attention mechanism obtains the features of different words in the text by weighting the text sequence, so as to obtain the critical iinformation in the text to the maximum extent. Attn-BiLSTM model adds attention layer to original BiLSTM model and carries out a weighted calculation for BiLSTM output. Combining the advantages of attention mechanism and BiLSTM model, this model can highlight the features of high weight in corpus and improve the analytical ability of the model. The corpus is vectorized by word vector model, and the semantic features of the corpus were obtained by input Attn-BiLSTM model. The semantic features are weighted by attention mechanism to obtain the relatively important features, and the public sentiment distribution is predicted by the activation function layer.

## 4. Data Analysis

### 4.1. Descriptive Analysis

This study split the “Double Reduction Policy” event into four stages, which include the generation stage, outbreak stage, fading stage, and secondary outbreak stage. Among them, July 1, 2021–August 12, 2021 was the generation stage, August 13, 2021–September 5, 2021 was the outbreak stage, September 6, 2021–October 6, 2021 was the fading stage, and October 7, 2021–October 18, 20201 was the secondary outbreak stage. We construct multiple time-series datasets, and regard the segmentation of public opinion evolution as the temporal dimension, and the amount of microblog posts in different regions as *x*-axis. The visualization is shown in Figure 2.

The distribution of microblogs represents the trend of public attention. It could be found that the whole attention of public sentiment spreads from coastland and central provinces (such as Jiangsu, Guangdong, Zhejiang, Shanghai, Shandong, Henan, Anhui, Hubei, and Liaoning) to central and western provinces. During the generation stage, the provinces (municipalities) with the highest attention are Jiangsu, Chongqing, Guangdong, and Henan. When the “Double Reduction Policy” is implemented actually, the public sentiment also developed into the outbreak stage. Netizens show much more enthusiastic about this policy. In the fading stage, the public attention gradually spread to the central and western provinces, and the percentage of microblog posts in those provinces began rising. In the secondary outbreak stage, the attention returned to the developed coastal areas and the central education provinces.

### 4.2. Clustering Analysis

The event extraction includes the trigger words recognition and time elements extraction. The “industry impact,” “Institutional supervision,” “public feedback,” “policy implement,” and the corresponding list of trigger words are generated by the LDA model and LTP. We use a script to filter the “dataset” by trigger words and obtain the body of microblogs under each topic event and the corresponding comment data as shown in Table 2.

The “Industry impact” covers the influence of “Double Reduction Policy” on the tutoring firms and the reverberations. The direct influences include the suspension, closure, bankruptcy, and refund. The “Institutional supervision” covers the regulatory statements, reporting and governance incidents of tutoring firms after the implementing of the “Double Reduction Policy.” The “Public feedback” covers the students' and their parents' reaction to the changes after the “Double Reduction Policy” was implemented, such as remedial classes, return to the classroom, quality education, and reduction of the burden. The reaction also includes their uncertainty about the future. The “Policy implement” covers the influence (job loss, career change) of the “Double Reduction Policy” on education practitioners (primary and secondary school teachers, teachers in training institutions).

### 4.3. Sentiment Analysis

In the research method section, this study designs 2 sentiment analysis method including sentiment vocabularies calculate algorithm and deep learning model. We compare the results of these two methods and finds out the algorithm method is faster than model, whereas the Attn-BiLSTM model could figure out some obscure sentiment text.  Table 3 shows the public sentiment analysis result based on Attn-BiLSTM, which reveals the public sentiment levels are polarized. In the lifecycle dimension, with the event development, the negative sentiment, disgust, raised to the peak in secondary outbreak stage, and the percentage of optimism plummeted to 0.11% at the same time. The cause of this phenomenon is related to the policy impacting on the tutor firms. In this study, government policy announcements and media reports are labeled as “beauty” (because the sentiment category of “beauty” includes trust element). And in the sample of the “beauty” sentiment category corpus indicate that most policy interpretations, announcements, and reports are classified in this category. The sentiments of “sadness” and “fear” also show higher in front and lower behind. We suppose that is related to the fact that netizens do not understand the policy when it was promulgated. The public are not optimistic about the future of education.

As shown in Table 4, in the topic of “industry impact,” the public sentiment is correlated with their social role (teachers in tutoring firms, students, and parents) significantly. More than half of the netizens show positive emotional feedback on the “Double Reduction Policy” during the generation stage, outbreak stage, and fading stage. The “Double Reduction Policy” and the introduction of substantive measures around the tutoring firms caused a significant impact. The suspension, closure, and bankruptcy of tutoring institutions are reflected in the disgust among netizens during the outbreak stage, fading stage, and secondary outbreak stage. This study filters the relevant microblogs and figures out that the main reason is the institutions' capital chain broke cased the inability to settle teachers' class fees and salaries, as well as parents' prepaid tuition fees after.

As shown in Table 5, in the topic of “Institutional supervision,” the transformation of public sentiment becomes more complicated. The “disgust” and “beauty” take up the most significant proportion. With the beginning of term, the public sentiment evolute into the outbreak stage. The sentiment of “disgust” shorts up by 74.9% and remains at a high level. The sentiment of “beauty” dropped from 32.5% in the generation stage to 2.46% in the second outbreak stage. During the generate stage, most netizens hold a wait-and-watch attitude. The microblogs in that stage indicate the netizens do not fully recognize the impact of supervision. Some netizens even generate the feelings of expectation. However, after the implementation of the policy, the counseling institutions fled, and the teachers and parents failed to protect their rights, resulting in a sharp increase of “disgust” among netizens, requiring the government to strengthen the supervision of counseling institutions.

As shown in Table 6, in the topic of “public feedback,” netizens gave good emotional feedback in the first three stages, and the worries and concerns are various in different periods. In the generate stage, it focuses on the fear about the tutoring after schools, academic pressure, expecting a rapid transformation of education through the policy implement. In the outbreak and fading stages, it focuses on the education system perfection, artificial intelligence supports education, and returning to school. In these stages, a certain number of parents and students represent “disgust,” “fear,” “sorrow,” and other negative sentiment about the teaching content, the decrease of schoolwork pressure, the extracurricular life, and their future. Netizens in different regions and social stratums might express completely opposite sentiment comments.

As shown in Table 7, in the topic of “Policy implement,” disgust and beauty are the most fluctuating sentiments. For the generate stage is in Chinese summer holiday, teachers in schools respond with beauty sentiment. Some teachers of tutoring institutions represent “sadness” emotions about the future of the tutoring industry. In September, students are back to schools, the “Double Reduction Policy” has the opposite impact on tutoring firms and schools. Tutoring institutions have shut down classes. In respond to the “Double Reduction Policy,” schools reduced the burden or over-learning by using the materials beyond the teaching syllabus.

These pressures are transferred to the teachers, students, and parents eventually, and the network public sentiments are diverging. Teachers lost their employment in tutoring firms are becoming fear, sadness, and disgust about their futures. They turn to achieve for jobs in the government system. Similarly, teachers in schools are required to take up “after-school service,” which has a great impact on the teachers accustom lives. The teachers represent resistance and other disgust sentiment. Parents and students are worried about the results of the exams after the policy implementation. These above negative emotions come to a climax in the secondary outbreak stage.

Based on the network public sentiment analysis result, this study reveals four topics in four stages, respectively. These topics include “industry impact,” “institutional supervision,” “public feedback,” and “policy implementation”. In the whole distribution of sentiments, the beauty and disgust emotions account for the highest proportion, this appearance indicates a trend of polarization. In the lifecycle dimension, network public sentiment evolution shows a trend of optimism during the generate stage, pessimism during the fading and secondary outbreak stage. During the secondary outbreak stage, in the topic of “institutional supervision,” a great deal of institutions shut down, and the follow-up teachers and parents refund rights are not favorable, which pushed the disgust proportion to the peak. The main body of this public sentiment is students, parents, teachers of tutoring firms and schools, and official accounts. This study reveals some common characteristics in the sentiment's evolution of students, parents, and teachers. The closure of counseling institutions obstructs the recovery of tuition fees and labor fees, which generate disgust emotion. The confusion and disappointment of personal development (entering high schools, teachers transforming) generates sadness and fear emotions. School teachers mostly expressed their discomfort with the increased workload and the break in their habits.

As an important policy that will influence the education industry future development, “Double Reduction Policy” should be promulgated and promoted with full consideration of the pressure of public opinion brought about by the policy. The official accounts should reasonably guide the development of public opinion at all stages of the development of public opinion. The public sentiment supervision department should intervene in a timely manner to guide the reasonable development of public sentiment. However, this study reveals that the official accounts (education departments and experts) do not pay enough attention to these issues, and the voice is controlled by opinion leaders and self-media accounts. In the analysis of the corresponding corpus, we find the expression of these education opinion leaders and self-media accounts are mostly negative, such as “panic,” “boredom,” “blame,” and “doubt”. Due to the lack of official guidance, the rational and positive voices in the microblogs and comments are also covered by those accounts. Based on this analysis, we present a sentiment guidance strategy, as shown in Figure 3. This strategy focuses on the organization guidance in different sentiment life stages. In normal sentiment evolution, the netizens' opinion is influenced by the opinion leaders (KOL) and self-media accounts significantly. These sentiments are reflected on the emotion relevant multimodal corpus. So that this strategy supposes the organization should pay more attention on the corresponding vocabularies propagation channel, especially between the KOL and netizens. This strategy emphasis the generate, outbreak, and secondary outbreak stages. Especially in the last stage, the organization should supervise and guide relevant sentiments to avoid secondary public sentiment.

## 5. Discussion and Conclusion

This study analyzes the impact of “Double Reduction Policy” on public sentiment in the microblog platform. The interpretation could support governments to accurately grasp the situation of network public sentiment and do a good job of propaganda and public opinion guidance in a scientifically and efficiently way. First, 10,155 news items and 22,463 comments related to the “Double Reduction Policy” are retrieved from the microblog platform, and the LDA topic clustering model combined with LTP is used to cluster four thematic events including “industry impact,” “institutional supervision ” “public feedback,” “policy implement,” and the corresponding list of trigger words. Based on the sentiment dictionary and modifier dictionary, the sentiment score is calculated. The sentiment distribution of Internet users is obtained by the Attn-BiLSTM model. A data mining is conducted based on the sentiment distribution, geographical distribution, and corpus text. Based on the sentiment analysis results, this study figures out a response strategy based on the sentiment lifecycle. We suppose the administration should pay more attention in the sentiment generate and outbreak stage. In addition, we also believe the secondary outbreak stage should be spent more attention. During the sentiment guidance, more attention should be paid on the negative emotion vocabulary, since these words could inspire more branch public sentiment. The interpretation based on this sentiment events could support the government's public opinion management. The government should guide the network sentiment at the generate stage, and track the whole lifecycle of the event to confirm the voice right. This study also has some shortcomings, such as the pretrained language model used in this paper is a static word vector model, which is not perfect and may affect the sentiment classification results. The above problems will be added in the subsequent research.

## Figures and Tables

**Figure 1:** Construction of Attn-BiLSTM model [43].

**Figure 2:** Microblogs post volume in different provinces.

**Figure 3:** Sentiment guidance strategy.

**Table 1:** Data cleaning rules.

Id	Rules	Note
1	Mid (the microblog index) repeat	A single microblog post might corresponding with multitopics
2	Special format (HTML, reply symbol, @, emojis, topic symbol)	HTML and reply symbols do not contain substantial information, and emojis might affect the accuracy of model training
3	Stop words	High-frequency words

**Table 2:** Topic events and trigger words.

Id	Topic event	Trigger words	Posts	Comments
1	Industry impact	Refunds; claims; tuition; runaway; rights; explosions; fees; training; collapse; stopping classes; bankruptcy; refunds; vipkid; complaints	2814	8345

2	Institutional supervision	Irregularities; regulation; schooling; investigation; reporting; supervision; registration; governance; management	1940	2238

3	Public feedback	Secondary school exams; remedial classes; reduce the burden; return; high school exams; start of school; quality; inside the volume; parents; children; semester	2140	5364

4	Policy implement	Unemployment; transformation; service; off duty; hosting; work; how; industry; market; pressure	1048	3492

**Table 3:** The distribution of public sentiment.

Sentiment categories	Generate stage (%)	Outbreak stage (%)	Fading stage (%)	Secondary outbreak stage (%)
Anger	0.08	0.31	0.14	0.11
Disgust	32.75	45.28	58.10	80.34
Fear	2.50	1.87	1.72	0.45
Optimism	55.75	44.90	32.66	15.14
Beauty	1.33	1.46	0.38	0.11
Sadness	5.67	3.46	2.92	0.79
Shock	1.92	2.72	4.09	3.05

**Table 4:** The distribution of public sentiment in the topic of “industry impact”.

Sentiment categories	Generate stage (%)	Outbreak stage (%)	Fading stage (%)	Secondary outbreak stage (%)
Anger	0.00	0.45	0.21	0.00
Disgust	26.46	39.44	45.45	63.93
Fear	3.61	1.89	1.93	0.55
Optimism	59.97	48.97	42.99	31.15
Beauty	1.72	1.53	0.64	0.00
Sadness	6.19	4.76	4.92	2.19
Shock	2.06	2.96	3.85	2.19

**Table 5:** The distribution of public sentiment in the topic of “institutional supervision”.

Sentiment categories	Generate stage (%)	Outbreak stage (%)	Fading stage (%)	Secondary outbreak stage (%)
Anger	0.00	0.20	0.00	0.21
Disgust	52.50	74.90	85.23	94.05
Fear	3.33	1.78	1.82	0.00
Optimism	32.50	16.01	5.81	2.46
Beauty	0.00	0.59	0.12	0.00
Sadness	7.50	1.58	1.21	0.21
Shock	4.17	4.94	5.81	3.08

**Table 6:** The distribution of public sentiment in the topic of “public feedback”.

Sentiment categories	Generate stage (%)	Outbreak stage (%)	Fading stage (%)	Secondary outbreak stage (%)
Anger	0.29	0.31	0.28	0.00
Disgust	39.26	38.79	48.28	26.12
Fear	1.15	1.94	1.51	1.16
Optimism	52.15	51.79	43.33	63.41
Beauty	0.86	1.94	0.41	1.16
Sadness	5.44	3.79	3.44	2.33
Shock	0.86	1.43	2.75	5.81

**Table 7:** The distribution of public sentiment in the topic of “policy implement”.

Sentiment categories	Generate stage (%)	Outbreak stage (%)	Fading stage (%)	Secondary outbreak stage (%)
Anger	0.00	0.00	0.00	0.00
Disgust	26.17	39.08	49.88	72.09
Fear	0.67	1.72	1.43	1.55
Optimism	66.44	54.60	43.94	24.03
Beauty	2.01	1.15	0.24	0.00
Sadness	2.68	1.15	0.95	0.00
Shock	2.01	2.30	3.56	2.33

## Data Availability

The data used to support the findings of this study can be obtained from the corresponding author upon request.
